RETRACTED

# Arnebin-1 promotes angiogenesis by inducing eNOS, VEGF and HIF-1α expression through the PI3K-dependent pathway

**DOI:** 10.3892/ijmm.2015.2292

**Published:** 2015-07-22

**Authors:** ZHI ZENG, WEN-DONG HUANG, QI GAO, MEI-LING SU, YONG-FEI YANG, ZHAO-CHUN LIU, BANG-HAO ZHU

**Affiliations:** Department of Pharmacology, Cardiac and Cerebral Vascular Research Centre, Zhongshan School of Medicine, Sun Yat-sen University, Guangzhou, Guangdong 510080, P.R. China

**Keywords:** arnebin-1, angiogenesis, hypoxia-inducible factor, vascular endothelial growth factor, endothelial nitric oxide synthase, diabetic wound, phosphatidylinositol 3-kinase-dependent pathway

## Abstract

Arnebin-1, a naphthoquinone derivative, plays a crucial role in the wound healing properties of Zicao (a traditional wound healing herbal medicine). It has been noted that Arnebin-1, in conjunction with vascular endothelial growth factor (VEGF), exerts a synergistic pro-angiogenic effect on human umbilical vein endothelial cells (HUVECs) and accelerates the healing process of diabetic wounds. However, the mechanisms responsible for the pro-angiogenic effect of arnebin-1 on HUVECs and its healing effect on diabetic wounds have not yet been fully elucidated. In this study, in an aim to elucidate these mechanisms of action of arnebin-1, we investigated the effects of arnebin-1 on the VEGF receptor 2 (VEGFR2) and the phosphoinositide 3-kinase (PI3K)-dependent signaling pathways in HUVECs treated with VEGF by western blot analysis. The pro-angiogenic effects of arnebin-1 on HUVECs, including its effects on proliferation and migration, were evaluated by MTT assay, Transwell assay and tube formation assay *in vitro*. The expression levels of hypoxia-inducible factor (HIF)-1α, endothelial nitric oxide synthase (eNOS) and VEGF were determined by western blot analysis in the HUVECs and wound tissues obtained from non-diabetic and diabetic rats. CD31 expression in the rat wounds was evaluated by immunofluorescence staining. We found that the activation of the VEGFR2 signaling pathway induced by VEGF was enhanced by arnebin-1. Arnebin-1 promoted endothelial cell proliferation, migration and tube formation through the PI3K-dependent pathway. Moreover, Arnebin-1 significantly increased the eNOS, VEGF and HIF-1α expression levels in the HUVECs and accelerated the healing of diabetic wounds through the PI3K-dependent signaling pathway. CD31 expression was markedly enhanced in the wounds of diabetic rats treated with arnebin-1 compared to the wounds of untreated diabetic rats. Therefore, the findings of the present study indicate that arnebin-1 promotes the wound healing process in diabetic rats by eliciting a pro-angiogenic response.

RETRACTED

## Introduction

In developed countries, a major cause of hospital admissions for patients with diabetes is chronic diabetic foot ulcers, which are a common symptom of diabetes and often result in pain and a lower quality of life (1). It has been reported that 15% of all patients with diabetes develop chronic diabetic foot ulcers, and in 84% of cases, this leads to amputation (2,3). There is, as yet, no widely available effective treatment strategy for diabetic foot ulcers. Consequently, novel effective treatment strategies for this chronic complication of diabetes are urgently required (4,5).

Relative hypoxia is a critical stimulus for normal wound healing, and the major cause of impaired wound healing in patients with diabetes may be an impaired response to hypoxia (6). Hypoxia-inducible factor (HIF)-1, a heterodimer, includes two subunits, a hypoxia-stabilized α-subunit (HIF-1α) and a constitutively expressed β-subunit (HIF-1β), which plays an important role as a master regulator of oxygen homeostasis. Under hypoxic conditions, HIF-1α is stabilized and moves towards the nucleus, dimerizing with HIF-1β. Subsequently, the dimer binds to a hypoxia response element (HRE), which appears on several genes that are responsible for cell survival during hypoxia (7). HIF-1α mediates the expression of numerous pro-angiogenic growth factors, such as vascular endothelial growth factor (VEGF), as well as the recruitment of endothelial progenitor cells to sites of vascularization through endothelial nitric oxide synthase (eNOS) and cell motility (8–10).

Diabetic foot ulcers heal slowly due to impaired neovascularization in response to tissue ischemia (11). Multiple growth factors and cytokines are involved in the formation of new blood vessels during wound healing. Of all the known pro-angiogenic molecules, VEGF is the most important mediator that promotes angiogenesis (12–14). It has been previously reported that the expression of VEGF is attenuated in diabetes (15). VEGF exerts major biological effects by binding with and stimulating its receptors. Among these, VEGF receptor 2 (VEGFR2) is an important receptor that transduces VEGF-activated signaling in endothelial cells. The activation of VEGFR2 leads to the phosphorylation of specific downstream signal transduction mediators, including protein tyrosine kinase, extracellular signal-regulated kinase (ERK) and focal adhesion kinase (FAK). As previously demonstrated, VEGFR2 signaling is necessary for the implementation of VEGF-induced vascular permeability, proliferation, migration and the sprouting of endothelial cells *in vitro* and neovascularization in wound healing (16–19).

RETRACTED

Although some therapeutic methods, such as gene therapy and treatment with recombinant growth factors have been used in an aim to promote angiogenesis, these methods are impeded by limitations, such as safety issues and high costs (20). A pharmaceutical method may thus be the most effective and advantageous method, particularly in terms of convenience, cost and safety. Zicao is a traditional herbal medicine used to promote wound healing that has been applied for hundreds of years in China (21). A survey of the published studies revealed that arnebin-1, a naphthoquinone derivative, plays a crucial role in the wound-healing properties of Zicao. A previous study demonstrated that arnebin-1 significantly accelerated both normal and hydrocortisone-impaired wound healing compared with the controls (22). In a recent study of ours, we also reported that arnebin-1 promoted the wound healing process in diabetic rats (23). Thus, arnebin-1 significantly accelerates the wound healing process; however, the specific mechanisms involved remain unknown, particularly those in relation to diabetic wounds.

Therefore, the aim of the present study was to investigate the mechanisms responsible for the pro-angiogenic effects of arnebin-1 on human umbilical vein endothelial cells (HUVECs), as well as those responsible for its healing effects on wounds of rats with alloxan-induced diabetes mellitus (DM). The effects of arnebin-1 on the phosphoinositide 3-kinase (PI3K)-dependent signaling pathway, VEGFR2 signaling and on the expression levels of eNOS, VEGF and HIF-1α *in vitro* were also determined. Moreover, to confirm the promoting effects of arnebin-1 on neovascularization in diabetic wounds, the protein expression levels of HIF-1α, eNOS, VEGF and CD31 were also determined in wound tissues from non-diabetic and diabetic rats.

## Materials and methods

### Materials

Arnebin-1 was purchased from Tokyo Chemical Industry Co. Ltd. (Tokyo, Japan), and recombinant human VEGF was from PeproTech Inc. (Rocky Hill, NJ, USA). Growth factor-reduced Matrigel basement membrane matrix was obtained from BD Biosciences (Bedford, MA, USA). Medium 199 (M199) and fetal bovine serum (FBS) were purchased from Gibco (Carlsbad, CA, USA). LY294002, a PI3K inhibitor, was purchased from Wako Pure Chemical Industries, Ltd. (Osaka, Japan). All other reagents utilized were purchased from Sigma Chemical Co. (St. Louis, MO, USA) unless otherwise specified.

### Cell culture

The isolation and culture of the HUVECs was carried out as previously described (21). Briefly, following digestion with 0.125% trypsin, the HUVECs were removed from human umbilical veins which were obtained following delivery. The HUVECs were removed from the umbilical veins following digestion with 0.125% trypsin and then cultured in M199 containing 20% FBS, 100 U/ml penicillin, 100 U/ml streptomycin and 50 U/ml heparin, supplemented with 2 mM L-glutamine, 1 mM sodium pyruvate and 5 ng/ml β-endothelial cell growth factor (β-ECGF) at 37°C in 5% CO_2_ in gelatin-coated culture flasks. Endothelial cells were identified by their morphology (cobblestone or mosaic-like appearance) after reaching confluence and by the presence of von Willebrand factor (data not shown). Passage 3–6 HUVECs were used in all the experiments. This study was approved by the Ethics Committee of Sun Yan-sen University (Guangzhou, China).

RETRACTED

### Cell proliferation assay

Cell proliferation was examined by mitochondrial MTT tetrazolium assay. The HUVECs were plated at 3×10^3^ cells/well in 96-well plates. Overnight, the HUVECs were pre-treated with or without LY294002 (2 *µ*M), and the medium was then replaced with the test medium supplemented with the vehicle [dimethyl sulfoxide (DMSO)] and arnebin-1 (10^−1^ *µ*M) with or without 1 ng/ml VEGF. After 24 h of incubation, the number of viable cells was detected using MTT reagent according to the manufacturer's instructions. In brief, 10 *µ*l MTT (5 mg/ml) was added to 100 *µ*l medium, and cultivated at 37°C for 4 h. After removing the supernatant, the formazan crystals were solubilized by the addition of DMSO. The absorbance (570 nm) of the medium was determined using a Biotek Elx-800 plate reader (BioTek Instruments, Inc., Winooski, VT, USA).

### Cell migration assay

Cell migration assay was performed using Transwell chambers as previously described (21). The bottom chamber of the device contained 600 *µ*l of the test medium. The HUVECs (5×10^4^ cells/well) were added to the upper chamber and cultured in M199 medium with 2% FBS. After 24 h of incubation, the non-migrated cells that were above the faces of the membranes were removed. The migrating cells were fixed with methanol for 15 min, and then stained with 0.1% crystal violet for 20 min. The membranes were then rinsed with 30% glacial acetic acid. Finally, the washing solution was examined at 540 nm for the counting of the number of HUVECs.

### Tube formation assay

To examine the pro-angiogenic effect Arnebin-1, we used the experimental *in vitro* Matrigel system, as previously described (23). Growth factor-reduced Matrigel basement membrane matrix was thawed on ice at 4°C overnight, and all pipettes and 96-well flat bottom plates were pre-cooled before use. The 96-well plates were coated with 50 *µ*l Matrigel per well for 30 min at 37°C. The HUVECs were seeded at 4×10^4^ cells per well in 100 *µ*l assay medium. After 16 h of incubation, tube-like structures were photographed using an inverted microscope (IX71; Olympus Corp., Tokyo, Japan). The total tube length was quantified using ImageJ software (NIH, Bethesda, MD, USA).

RETRACTED

### Western blot analysis

The HUVECs were lysed using protein lysis buffer and protease inhibitor cocktail. The protein concentrations of the cell lysates were quantified using a bicinchoninic acid assay (BCA) kit, and equal amounts of protein were separated by SDS-PAGE and then transferred onto polyvinylidene fluoride (PVDF) membranes (Millipore, Billerica, MA, USA). The membranes were blocked in 5% non-fat dried milk diluted with Tris-Buffered Saline Tween-20 (TBST; in mmol/l: Tris-HCl 20, NaCl 150, pH 7.5 nd 0.1% Tween-20) at room temperature for 1 h and probed overnight at 4°C with a polyclonal rabbit anti-phosphorylated (p-)VEGFR2 (#2478), a polyclonal rabbit anti-VEGFR2 (#9698), a polyclonal rabbit anti-p-Erk1/2, a polyclonal rabbit anti-Erk1/2, a polyclonal rabbit anti-p-FAK (#8556), a polyclonal rabbit anti-FAK (#13009), a polyclonal rabbit anti-p-Src (#5473), a polyclonal rabbit anti-Src (#2109), a polyclonal rabbit anti-PI3K (#4257), a polyclonal rabbit anti-p-PI3K (#3821), a polyclonal rabbit anti-Akt (#4691), a polyclonal rabbit anti-p-Akt (#4060), a polyclonal rabbit anti-p-mammalian target of rapamycin (mTOR; #2983), a polyclonal rabbit anti-p-mTOR (#2971; all from Cell Signaling Technology, Beverly, MA, USA), a polyclonal rabbit anti-proliferating cell nuclear antigen (PCNA; sc-7907), a polyclonal rabbit anti-eNOS (sc-654), a monoclonal rabbit anti-VEGF (sc-152; both from Santa Cruz Biotechnology Inc., Santa Cruz, CA, USA) or a monoclonal rabbit anti-HIF-1α antibody (NB-100-479; Novus Biologicals, Littleton, CO, USA), and then incubated for 2 h with anti-rabbit IgG (Santa Cruz Biotechnology Inc.). Incubation with polyclonal mouse β-actin antibody (#3700; 1:3,000 dilution; Cell Signaling Technology) or monoclonal mouse α-tubulin antibody (T5168; 1:1,000 dilution; Sigma) was used as the internal standard control. The proteins were visualized using ECL™ western blotting detection reagents (Amersham Biosciences Corp., Piscataway, NJ, USA). The densitometry of the bands was quantified using ImageJ 1.38X software.

### VEGF enzyme-linked immunosorbent assay (ELISA)

A Quantikine human VEGF ELISA kit (R&D Systems, Minneapolis, MN, USA) was used according to the manufacturer's instructions. Briefly, VEGF standards and the conditioned medium from the HUVECs were placed into wells overlaid with antibody specific for human VEGF. After binding with an VEGF enzyme-linked polyclonal antibody specific for VEGF, the absorbance was measured at 450 nm using a microplate reader. The VEGF concentration was evaluated (in pg/ml) with the standard curve and adjusted for protein concentrations.

RETRACTED

### In vivo experiments

#### Animals and induction of diabetes

All animal procedures were approved by the Laboratory Animal Center of Sun Yat-sen University. As previously described (23), male Sprague-Dawley (SD) rats (weighing 250–300 g) were kept in stainless steel cages under pathogen-free conditions. The rats were housed in a controlled environment with a constant temperature of 18–22°C and a 12-h light-dark cycle; the rats were allowed access to food and water *ad libitum*. The rats were allowed to acclimatize for 4 weeks before the experimental procedures commenced. The rats were fasted for 12 h and were injected intraperitoneally with alloxan monohydrate dissolved in normal saline at a double dose of 100 mg/kg every other day to induce diabetes. Following the administration of alloxan for 3 days, the fasting blood glucose (FBG) levels of the rats were measured using a glucometer. The rats exhibiting FBG levels >16.7 mmol/l were confirmed as diabetic rats for the purposes of our research. The FBG levels were monitored before and after the experiments. The animals were randomly divided into 4 groups (1 non-diabetic and 3 diabetic groups; n=6) as follows: i) the non-diabetic group: rats were administered distilled water for 7 days (non-diabetic group); ii) the first diabetic group: the diabetic animals received distilled water (diabetic group); iii) the second diabetic group: the diabetic animals received the vehicle (ointment without arnebin-1; DM-vehicle; D + V group); and iv) the third diabetic group: the diabetic animals were treated with arnebin-1 ointment (DM-arnebin-1; D + A group) for 7 days.

#### Preparation of the ointment

As described in a previous study of ours (23), ointment containing siritch (1.5 g), beeswax (5 g) and lard oil (0.15 g) was heated at 70–75°C to become solubilized, and 6.65 mg arnebin-1 (0.1%) was then added and mixed in. Finally, the mixture was stirred until it cooled to room temperature. This ointment was used as the test compound.

#### Experimental wounding

As previously described (23), SD rats were anesthetized with sodium pentothal (35 mg/kg, by intraperitoneal injection). The hair on the dorsal side of each rat was shaved, and the skin was sterilized with 70% ethanol. Full thickness cutaneous wounds were made with an 8-mm skin biopsy punch (World Precision Instruments, Sarasota, FL, USA) under aseptic conditions. Three wounds were made on the dorsal surface of the diabetic rats, and one wound was made on the non-diabetic rats. The diameters of the wounds ranged between 7.5 and 9 mm. Thereafter, the animals were individually caged.

RETRACTED

#### Drug administration

As stated above, each diabetic rat had 3 wounds on the dorsal surface and the non-diabetic rats had 1 wound. In the D + V group, only wounds on the top of the dorsal side were treated with only the vehicle base (without the test compound). In the diabetic group, only wounds near the tail were treated with distilled water. In the D + A group, only wounds in the middle were treated with arnebin-1 (0.1% ointment). Thus, in each group of rats, a different wound area was treated. The wounds at the top served as the vehicle controls for the treated wounds. The test compound ointment and the vehicle were applied every other day, in quantities sufficient to cover the wounds with a thin layer. All the treatments were continued until the day of sacrifice. The rats were sacrificed with the use of an intraperitoneal injection of an overdose of barbiturate.

#### Tissue collection

The rats were anesthetized with an overdose of pentobarbital (200 mg/kg, injected intraperitoneally) on day 7 post-wounding. The wound and a margin of approximately 5 mm of unwounded skin was excised. These wound tissues were snap-frozen in liquid nitrogen until they were processed for protein isolation.

#### Western blot analysis

In order to measure the levels of PCNA, CD31, HIF-1α, VEGF and eNOS in the tissue, wounds treated with arnebin-1 or the vehicle were harvested on day 7 post-wounding. Following excision, the tissues were homogenized in lysis buffer. The VEGF, eNOS and HIF-1α expression levels were determined by western blot analysis as described above.

#### Immunofluorescence staining for CD31

Wound samples, taken on day 7, were embedded in paraffin and frozen in liquid nitrogen immediately for immunofluorescence. To assess new blood vessel formation, vessel density was estimated after staining for CD31. Serial 6-*µ*m frozen sections were incubated with primary antibodies for CD31 (1:100; 550274; BD Biosciences) at 4°C overnight. Subsequently, the sections were washed with phosphate-buffered saline (PBS) 3 times and incubated with goat anti-rat IgG-Cy3 (1:200; A0507; Beyotime Institute of Biotechnology, Shanghai, China) for 1 h at 37°C. Hoechst 33342 dye (C1026; Beyotime Institute of Biotechnology) was used to stain the nuclei for 3–5 min at room temperature. The sections were examined and photographed under a fluorescence microscope (IX71; Olympus Corp.). The number of CD31-positive vessels was determined across 5 non-consecutive tissue sections for each wound.

#### Statistical analysis

All statistical analyses were performed using GraphPad Prism 5.0 (GraphPad Software, Inc., USA). Data for each study parameter from each group are presented as the means ± standard error of the mean (SEM). Data from each group were statistically analyzed by one-way analysis of variance (ANOVA). Differences were considered statistically significant at P<0.05.

RETRACTED

## Results

### Effect of arnebin-1 on the proliferation of HUVECs

PCNA is a nuclear cell proliferation marker. To determine whether arnebin-1 promotes the proliferation of HUVECs, the PCNA levels were measured by western blot analysis. At concentrations ranging from 1×10^−3^ *µ*M to 10^−1^ *µ*M, arnebin-1 alone had no significant effect on the PCNA levels (Fig. 1B). However, in the presence of VEGF (1 ng/ml), arnebin-1 significantly increased the expression of PCNA in a concentration-dependent manner (Fig. 1C). Consistent with the results of our previous study (23), we found that arnebin-1 had no noticeable effect on cell viability and proliferation (as no changes were observed in PCNA expression), as evaluated by MTT assay in the test range, but had a synergistic effect with VEGF in that it promoted HUVEC proliferation (Fig. 5A).

### Arnebin-1 activates the VEGFR2 signaling pathway

It has been reported that VEGFR2 phosphorylation activates extensive downstream signaling substrates that are closely related to endothelial cell proliferation, migration and tube formation (30). To investigate whether arnebin-1 activates VEGFR2 and its downstream signaling molecules, we screened some elementary kinases related to the VEGFR2 signaling pathway. As shown in Fig. 2, arnebin-1 significantly increased the phosphorylation of VEGFR2, FAK, ERK and Src, induced by VEGF (1 ng/ml), in a concentration-dependent manner, which suggested that arnebin-1 exerted its pro-angiogenic effect by directly targeting VEGFR2 and subsequently activating the VEGFR2-induced downstream signaling cascade. These results are consistent with those of our previous study, which demonstrated that arnebin-1 promoted the proliferation, migration and tube formation of HUVECs in a concentration-dependent manner in the presence of VEGF (23).

### Arnebin-1 upregulates the expression levels of eNOS, VEGF and HIF-1α in HUVECs in a PI3K-dependent manner

Subsequently, we investigated the effects of arnebin-1 on the expression levels of eNOS and VEGF in HUVECs. At concentrations ranging from 1×10^−3^ *µ*M to 10^−1^ *µ*M, arnebin-1 significantly increased the protein expression of eNOS in the HUVECs in a concentration-dependent manner compared to the vehicle-treated (control) cells (Fig. 3A). Moreover, arnebin-1 at 10^−2^ and 10^−1^ *µ*M also markedly increased the expression and secretion of VEGF protein compared with the control group (Fig. 3B and C). Similarly, the expression of HIF-1α was also markedly upregulated by arnebin-1 (Fig. 3D). We further examined whether the upregulation of eNOS, VEGF and HIF-1α by arnebin-1 in HUVECs is mediated by its effect on the PI3K pathway. The protein expression of HIF-1α was markedly reduced by treatment with 2 *µ*M LY294002 1 h prior to stimulation with 10^−1^ *µ*M arnebin-1 (Fig. 3E). Similarly, the protein expression of eNOS, and the expression and secretion of VEGF protein, were also significantly decreased following pretreatment with 2 *µ*M LY294002 (Fig. 3F–H).

RETRACTED

We also investigated whether arnebin-1 has any effect on the PI3K/Akt/mTOR pathway, which functions upstream of eNOS, VEGF and HIF-1α. Following treatment for 24 h, arnebin-1 induced a marked increase in the protein expression levels of PI3K, Akt and mTOR in the HUVECs in a concentration-dependent manner (Fig. 4A–C). Moreover, in the HUVECs treated with arnebin-1 at various concentrations (10^−3^, 10^−2^ and 10^−1^ *µ*M) for 2 h, the phosphorylation levels of these 3 proteins were significantly increased in a concentration-dependent manner (Fig. 4D–F). Taken together, these results demonstrate that arnebin-1 regulates the expression of eNOS, VEGF and HIF-1α in HUVECs in a PI3K-dependent manner.

### Arnebin-1 promotes the proliferation, migration and tube formation of HUVECs through the PI3K-dependent pathway

In a previous study (23), we confirmed that arnebin-1 significantly promoted the proliferation, migration and tube formation of HUVECs in the presence of VEGF (1 ng/ml) in a concentration-dependent manner, with a maximal effect at 10^−1^ *µ*M. In the present study, we investigated the mechanisms responsible for these effects of arnebin-1. As shown in Fig. 5, the proliferation, migration and tube formation of the HUVECs were enhanced by stimulation with a low concentration of VEGF (1 ng/ml) compared with the controls. Moreover, arnebin-1 at 10^−1^ *µ*M and VEGF had a synergistic effect and markedly increased these processes compared with the cells treated with VEGF alone. However, when the HUVECs were pre-treated with LY294002, a PI3K inhibitor, the synergistic effects of arnebin-1 and VEGF on cell proliferation, migration and tube formation were abolished (Fig. 5). As was also shown, pre-treatment with LY294002 attenuated the increase in the expression levels of eNOS, VEGF and HIF-1α induced by arnebin-1 (Fig. 3). Collectively, these results suggest that arnebin-1 promotes the processes of endothelial cell proliferation, migration and tube formation which are associated with angiogenesis through the upregulation of eNOS, VEGF and HIF-1α in a PI3K-dependent manner.

RETRACTED

### In vivo wound healing experiments

#### Induction of diabetes

The mean FBG levels and body weight of the animals are presented in Table I. The body weights and FBG levels of the non-diabetic rats and diabetic rats were determined before and 3 days after the alloxan injection. The rats exhibited a 3-4-fold increase in FBG levels compared to the normal levels after the alloxan injection and a concurrent decrease in body weight, indicating that DM was successfully induced in the rats. On the 7th day post-wounding, the FBG levels remained >16.7 mmol/l. Topical therapy applied to the wounds of the rats did not have any effect on the FBG level over the course of study.

#### Effect of arnebin-1 on the expression of HIF-1α, eNOS and VEGF in diabetic wounds

To investigate the mechanisms through which neovascularization is promoted, following treatment with arnebin-1, we measured the *in vivo* expression level of HIF-1α and its target genes, VEGF and eNOS. Western blot analysis revealed that the protein expression levels of HIF-1α, eNOS and VEGF were markedly decreased in the diabetic wounds compared with the non-diabetic wounds (Fig. 6). No significant difference was observed in the levels of HIF-1α, eNOS and VEGF between the diabetic and vehicle-treated groups. However, the expression of HIF-1α was markedly increased in the diabetic wounds following treatment with arnebin-1 (Fig. 6A). Compared with the diabetic and vehicle-treated groups, a higher level of eNOS expression was observed in the arnebin-1-treated group (Fig. 6B). Similarly, arnebin-1 significantly increased the protein expression of VEGF on the 7th day (Fig. 6C). Taken together, these results indicate that arnebin-1 promotes neovascularization in the wounds of diabetic rats by upregulating the expression levels of HIF-1α, eNOS and VEGF.

#### Effect of arnebin-1 on neovascularization and diabetic wound healing

In *in vitro* experiments, we demonstrated that arnebin-1 and a low concentration of VEGF significantly increased the expression of PCNA, and that the administration of arnebin-1 without VEGF did not achieve the same result. *In vivo*, there was still a low level of VEGF in the diabetic wound tissues, and the localized application of arnebin-1 ointment to the wounds upregulated the expression of PCNA compared with the diabetic group the and vehicle-treated group (Fig. 7A), which was in accordance with our *in vitro* results. To determine the role of arnebin-1 in neovascularization in diabetic wounds, the expression of CD31, a biochemical marker of angiogenesis, was examined to analyze the effects of arnebin-1. In our previous study, using histological analysis, we demonstrated that diabetic wounds treated with arnebin-1 exhibited an increased capillary density on days 4 and 7 post-wounding (23). In the present study, following immunofluorescence staining with an anti-CD31 antibody for endothelial cells, positive staining was present in the wounds of the non-diabetic rats (Fig. 7B). This staining appeared to be markedly reduced in the wounds of the diabetic control animals and the vehicle-treated diabetic animals. We found that the number of CD31-positive blood vessels around the granulation-formation region was increased on the 7th day following treatment with arnebin-1. The results from quantitative analysis revealed that capillary density was significantly greater in the arnebin-1-treated group than the diabetic group (Fig. 7C). Moreover, the results of western blot analysis indicated that the protein level of CD31 was significantly increased following treatment with arnebin-1 compared with the other diabetic groups not treated with arnebin-1 (Fig. 7D).

RETRACTED

## Discussion

At present, diabetic wounds remain a considerable challenge in clinical practice, and current treatments are inadequate. Only 66% of diabetic wounds ultimately heal, and up to 28% result in amputation (24–26). Deficient angiogenesis has been noted in abnormal wound healing that leads to diabetic foot ulcers (27). The diabetic wound environment is characterized by a marked decrease in the pro-angiogenic and angiogenic growth factors which regulate angiogenesis (28). In a previous study, we examined the effects of arnebin-1 on wound closure in diabetic rats and confirmed that treatment with arnebin-1 significantly accelerated diabetic wound closure compared with the rats which received the vehicle or no treatment (23). In this study, we demonstrate that arnebin-1 is an effective inducer of neovascularization, as it upregulates HIF-1α expression. Arnebin-1 promoted angiogenesis by increasing the expression of VEGF, eNOS and HIF-1α in a PI3K-dependent manner. By employing a wound model of type I diabetes, we demonstrated that the topical application of arnebin-1 significantly accelerated the wound healing process by promoting the angiogenic response. Based on these discoveries, we suggest that the upregulation of HIF-1α is an important procedure in arnebin-1-induced neovascularization, which contributes to wound healing (Fig. 8).

At present, there is no effective topical drugs which can be applied in routine clinical practice to treat diabetic foot ulcers (29). Since the pathogenesis of diabetic foot ulcers is complex, the application of a growth factor, such as VEGF or PDGF is an ineffective approach to promoting the closure of diabetic wounds. Taking into consideration the significance of the formation of new blood vessels in tissue repair and regeneration, previous researchers have attempted to apply various growth factors to accelerate angiogenesis in damaged wounds (30,31). If one substance can continuously release several growth factors to simulate the natural micro-environment, it could potentially be an optimal treatment for wound healing. However, this is difficult to achieve due to technological limitations and the high cost involved, and as a result, the application of this treatment method is limited. New approaches to effectively accelerate the wound healing process of diabetic wounds are urgently required.

RETRACTED

HIF-1α is necessary for the wound healing process, and the entire process of normal wound healing is dependent on its expression (32). HIF-1α plays a critical role in cell motility and regulates the expression of numerous pro-angiogenic growth factors, such as VEGF and also plays a role in the recruitment of endothelial progenitor cells (33). In diabetics, insufficient angiogenesis in wound healing could be caused by the reduction in the expression of HIF-1α and its target molecules, such as VEGF (11,34,32). Therefore, upregulating HIF-1α expression is possibly a more effective treatment strategy than applying a single growth factor. Moreover, taking into consideration the convenience, inexpensive nature and safety of application, the most functional and useful way to increase HIF-1α expression is to adopt a pharmaceutical approach.

Arnebin-1 has previously been shown to promote angiogenesis both *in vitro* and *in vivo* (23); however, its exact mechanisms of action and functions remain to be elucidated. In this study, by applying an excisional wound-healing model of diabetes, we demonstrated in this study that arnebin-1 upregulates HIF-1α expression and activates many endogenous target molecules necessary for wound healing, such as eNOS and VEGF.

It has long been recognized that blood supply is an important factor in wound healing. VEGF plays an essential role in promoting the growth of new blood vessels in certain organ systems (35). Thus, it acts as a critical stimulus in the promotion of angiogenesis, which assists in the healing of diabetic foot ulcers. In our previous study, compared to the vehicle-treated wounds, significantly enhanced vascularization was observed in the arnebin-1-treated wounds (23). VEGF is well known as a major regulator of neovascularization in wound healing. However, increasing the concentration of VEGF does not consistently promote wound healing (36). This means that there is a limitation to using only VEGF, and indicates that sufficient wound repair requires a variety of factors. HIF-1α is a major transcription factor, which induces VEGF expression, as well as the epxression of multiple molecules that are essential for wound healing (37). In the present study, we noted that arnebin-1 significantly increased the protein expression of HIF-1α as well as that of eNOS and VEGF in diabetic wounds. eNOS functions as a homing signal to mobilize vascular endothelial progenitor cells, which are responsible for vasculogenesis, from distant locations and recruit them to the location of the injury (38). As a result, we suggest that treatment with arnebin-1 induces the expression of HIF-1α-target molecules and enhances vascularization by promoting angiogenesis and vasculogenesis.

RETRACTED

In our *in vitro* experiments, we identified that treatment with arnebin-1 resulted in the upregulation of HIF-1α expression in the HUVECs in a concentration-dependent manner. Arnebin-1 did not increase the protein expression levels of eNOS, VEGF and HIF-1α in the HUVECs when the cells were pre-tretaed with LY294002, a PI3K inhibitor. We also noted that arnebin-1 induced the expression of angiogenic factors through HIF-1α. According to our previous data (23), treatment with arnebin-1 with low levels of VEGF stimulated endothelial cell function *in vitro* and markedly induced cell proliferation, migration and tube formation. In the present study, we observed that arnebin-1 promoted tube formation in HUVECs in a concentration-dependent manner. We also discovered that the arnebin-1-induced cell proliferation, migration and tube formation were PI3K-dependent. The effects induced by arnebin-1 were significantly inhibited by the suppression of the PI3K pathway which also inhibited HIF-1α expression.

VEGFR2 signaling is necessary for vascular endothelial cells to function. The main autophosphorylation site of VEGFR2 is tyrosine (Tyr)1175, and its phosphorylation initiates the downstream signaling events in endothelial cells (39). The mitogen-activated protein kinase (MAPK)/ERK cascade and the proliferation of endothelial cells are activated by the phosphorylation of Tyr1175 of VEGFR2, which also mediates the VEGF-induced activation of Src-mediated vascular permeability and cell migration (40,41). However, the activation of FAK through VEGFR2 has also been shown to be involved in VEGF-induced migration (42–44). In the present study, by directly increasing VEGFR2 phosphorylation, arnebin-1 subsequently promoted the activation of the ERK, FAK and Src signaling pathways and increased cellular activity, which were closely related to the upregulation of VEGF in HUVECs. These results suggest that arnebin-1 promotes angiogenesis through autocrine mechanisms.

eNOS activity has two important functions: it mobilizes endothelial progenitor cells from bone marrow to peripheral blood, and induces ischemia-induced vascularization (45). Since the PI3K/Akt/eNOS pathway plays a key role in the process of endothelial progenitor cell mobilization and homing (46), the results of the present study provide further insight into the effects of arnebin-1 on this pathway in HUVECs. Treatment with arnebin-1 markedly increased the protein expression levels of PI3K, Akt and eNOS, indicating the activation of the PI3K/Akt/eNOS pathway. Moreover, we noted that this pathway was stimulated by arnebin-1, and that the expression of HIF-1α was inhibited by LY294002. These results indicate that the PI3K/Akt/eNOS pathway mediates arnebin-1-induced HUVEC angiogenesis in a PI3K-dependent manner.

RETRACTED

In conclusion, based on the outcomes of the present study, and in conjunction with our previous data (23), we confirmed that arnebin-1 markedly promotes the angiogenesis of HUVECs *in vitro* and that the topical application of arnebin-1 ointment accelerates the wound healing process in type I diabetic rats by inducing the expression levels of eNOS, VEGF and HIF-1α through the PI3K-dependent signaling pathway. Topical treatment with arnebin-1 ointment may thus be considered a novel therapeutic stratety for diabetic foot ulcers. Clinical tests are warranted to determine whether treatment with arnebin-1 can promote wound healing in patients with diabetes. The exact effects of arnebin-1 on fibroblasts and keratinocytes remain also to be investigated.

## Figures and Tables

**Figure 1:** (A) Structure of arnebin-1 [5,8-dihydroxy-2-(1′-b,b-dimethylaryoxy-4′-methylpent-3-enyl)-1,4-naphthoquinone]. (B) Human umbilical vein endothelial cells (HUVECs) were treated with arnebin-1 only at various concentrations for 24 h. Cell lysates were subjected to western blot analysis. Upper panel shows representative blots of the protein expression of proliferating cell nuclear antigen (PCNA). Lower panel shows the quantification of the PCNA protein level. (C) The HUVECs were treated with arnebin-1 at various concentrations in the absence or presence of vascular endothelial growth factor (VEGF; 1 ng/ml) for 24 h. Cell lysates were subjected to western blot analysis. Upper panel shows representative blots of the protein expression of PCNA. Lower panel shows the quantification of the PCNA protein level. α-tubulin was used as a loading control. Bars represent the means ± SEM. ^*^P<0.05 vs. control; ^#^P<0.05 vs. VEGF-treated group. Control, vehicle-treated group.

**Figure 2:** Arnebin-1 promotes vascular endothelial growth factor (VEGF) receptor 2 (VEGFR2) kinase activity and its downstream signaling molecules. (A) Arnebin-1 increased the phosphorylation of VEGFR2 induced by VEGF in human umbilical vein endothelial cells (HUVECs). Total protein was isolated and subjected to western blot analysis. Upper panel shows representative blots of the protein levels of phosphorylated (p-)VEGFR2 and total (t-)VEGFR2 proteins. Lower panel shows the quantification of the p-VEGFR2 protein level. (B–D) Arnebin-1 also increased VEGFR2-mediated protein kinase activation of focal adhesion kinase (FAK), extracellular signal-regulated kinase (Erk) and Src. (B) Upper panel shows representative blots of the protein levels of p-FAK and t-FAK. Lower panel shows the quantification of the p-FAK protein level. (C) Upper panel shows the representative blots of the levels of p-Erk and t-Erk proteins. Lower panel shows the quantification of the p-Erk protein level. (D) Upper panel shows representative blots of the protein levels of p-Src and t-Src proteins. Lower panel shows the quantification of the p-Src protein level. (E) Diagram of signaling pathways involved in arnebin-1-induced angiogenesis. α-tubulin was used as a loading control. Bars represent the means ± SEM. ^*^P<0.05 vs. control; ^#^P<0.05, ^##^P<0.01 vs. VEGF-treated group. Control, vehicle-treated group.

RETRACTED

**Figure 3:** The expression levels of endothelial nitric oxide synthase (eNOS), vascular endothelial growth factor (VEGF) and hypoxia-inducible factor (HIF)-1α were increased by arnebin-1 in a phosphoinositide 3-kinase (PI3K)-dependent manner. (A–C) Human umbilical vein endothelial cells (HUVECs) were treated with arnebin-1 only at various concentrations (10^−3^, 10^−2^ and 10^−1^ *µ*M) for 24 h. Cell lysates were subjected to western blot analysis. (A) Upper panel shows representative blots of the protein level of eNOS. Lower panel shows the quantification of the eNOS protein level. (B) Upper panel shows representative blots of the protein level of VEGF. Lower panel shows the quantification of the VEGF protein level. (C) The secretion level of VEGF in the culture supernatants was determined by ELISA. (D) Upper panel shows representative blots of the protein level of HIF-1α. Lower panel shows the quantification of the HIF-1α protein level. (E–H) HUVECs were treated with or without LY294002 for 1 h, and then stimulated with arnebin-1 in the presence or absence of VEGF for 24 h. (E) Upper panel shows representative blots of the protein level of HIF-1α. Lower panel shows the quantification of the HIF-1α protein level. (F) Upper panel shows representative blots of the protein level of eNOS. Lower panel shows the quantification of the eNOS protein level. (G) Upper panel shows representative blots of the protein level of VEGF. Lower panel shows the quantification of the VEGF protein level. (H) The secretion level of VEGF in the culture supernatants was determined by ELISA. Bars represent the means ± SEM. ^*^P<0.05, ^**^P<0.01 vs. control; ^#^P<0.05, ^##^P<0.01 vs. Arnebin-1-treated groups. Control, vehicle-treated group.

RETRACTED

**Figure 4:** The effect of arnebin-1 on the phosphoinositide 3-kinase (PI3K) pathway. (A–C) Human umbilical vein endothelial cells (HUVECs) were treated with arnebin-1 only, at various concentrations (10^−3^, 10^−2^ and 10^−1^ *µ*M) for 24 h. Cell lysates were subjected to western blot analysis. (A) Upper panel shows representative blots of the protein level of total (t-)PI3K. Lower panel shows the quantification of the t-PI3K protein level. (B) Upper panel shows representative blots of the protein level of t-Akt. Lower panel shows the quantification of the t-Akt protein level. (C) Upper panel shows representative blots of the protein level of t-mTOR. Lower panel shows the quantification of the t-mTOR protein level. (D–F) HUVECs were treated with arnebin-1 only at various concentrations (10^−3^, 10^−2^ and 10^−1^ *µ*M) for 2 h. Cell lysates were subjected to western blot analysis. (D) Upper panel shows representative blots of the protein level of phosphorylated (p-)PI3K and t-PI3K. Lower panel shows the quantification of the p-PI3K/t-PI3K protein level. (E) Upper panel shows representative blots of the protein level of p-Akt and t-Akt. Lower panel shows the quantification of the p-Akt/t-Akt protein level. (F) Upper panel shows representative blots of the protein level of p-mTOR and t-mTOR. Lower panel shows the quantification of the p-mTOR/t-mTOR protein level. Bars represent the means ± SEM. ^*^P<0.05, ^**^P<0.01 vs. control. Control, vehicle-treated group.

**Figure 5:** Hypoxia-inducible factor (HIF)-1α is essential for arnebin-1-induced (A) cell proliferation, (B and C) cell migration and (D–E) tube formation of human umbilical vein endothelial cells (HUVECs) in the presence of vascular endothelial growth factor (VEGF). HUVECs were treated with or without LY294002 (2 *µ*M) for 1 h, and then stimulated with arnebin-1 (10^−1^ *µ*M) in the presence or absence of VEGF (1 ng/ml) for 24 h. (A) Cell proliferation was assessed by MTT assay. HUVECs were treated with or without LY294002 (2 *µ*M) for 1 h, and then stimulated with arnebin-1 (10^−1^ *µ*M) in the presence or absence of VEGF (1 ng/ml) for 8 h. (B and C) Cell migration was assessed by Transwell assay. HUVECs were treated with or without LY294002 (2 *µ*M) for 1 h, and then stimulated with arnebin-1 (10^−1^ *µ*M) in the presence or absence of VEGF (1 ng/ml) for 12 h. (D–E) HUVECs were plated on Matrigel to form tubular structures. Bars represent the means ± SEM. ^*^P<0.05, ^**^P<0.01 vs. control; ^#^P<0.05, ^##^P<0.01 vs. VEGF-treated group; and P<0.05 vs. VEGF + Arnebin-1-treated group. Control, vehicle-treated group.

RETRACTED

**Figure 6:** Effects of arnebin-1 on the hypoxia-inducible factor (HIF)-1α, vascular endothelial growth factor (VEGF) and endothelial nitric oxide synthase (eNOS) expression levels in diabetic rats. (A–C) Effects of arnebin-1 on the protein expression levels of HIF-1α, VEGF and eNOS. (A) Upper panel shows representative blots of the protein level of HIF-1α. Lower panel shows the quantification of the HIF-1α protein level. (B) Upper panel shows representative blots of the protein level of eNOS. Lower panel shows the quantification of the eNOS protein level. (C) Upper panel shows representative blots of the protein level of VEGF. Lower panel shows the quantification of the VEGF protein level. Bars represent the means ± SEM. ^*^P<0.05, ^**^P<0.01 vs. non-diabetic rats; ^#^P<0.05, ^##^P<0.01 vs. diabetic rats. n=6 for each group. D+V, diabetic rats treated with the vehicle; D+A, diabetic rats treated with arnebin-1.

**Figure 7:** Effects of arnebin-1 on proliferation and neovascularization in diabetic rats. (A) Effects of arnebin-1 on the expression levels of proliferating cell nuclear antigen (PCNA), a nuclear cell proliferation marker. Upper panel shows representative blots of the protein level of PCNA. Lower panel shows the quantification of the PCNA protein level. (B) Effects of arnebin-1 on wound vascularity. Wound sections were stained with an anti-CD31 antibody and detected with Cy3 (red). Representative immunofluorescence images of wound samples on day 7 after treatment. Immunostaining for CD31-positive blood vessels (red) was performed to show vasculature in wounds, and nuclei (blue) were counterstained with Hoechst 33342. (C) Quantitative analysis of CD31-positive blood vessels in each section. Results are expressed as the number of vessels per high-power field. (D) Effects of arnebin-1 on the expression levels of CD31. Upper panel shows representative blots of the protein level of CD31. Lower panel shows the quantification of the CD31 protein level. Bars represent the means ± SEM. ^*^P<0.05, ^**^P<0.01 vs. non-diabetic rats; ^##^P<0.01 vs. diabetic rats. n=6 for each group. D+V, diabetic rats treated with the vehicle; D+A, diabetic rats treated with arnebin-1.

**Figure 8:** Schematic diagram of the mechanisms through which arnebin-1 promotes vascularization and wound healing. Arnebin-1 treatment leads to the accumulation of hypoxia-inducible factor (HIF)-1α, and the consequent upregulation of VEGF and endothelial nitric oxide synthase (eNOS). The expression of HIF-1α target genes in turn promotes neovascularization in diabetic wounds through angiogenesis and vasculogenesis.

RETRACTED

**Table I:** Effects of arnebin-1 on body weight and blood glucose.

Factors	Non-diabetic rats (n=6)	Diabetic rats 3 days after injection (n=6)	Non-diabetic rats 7 days post-wounding (n=6)	Diabetic rats 7 days post-wounding (n=6)
Body weight (g)	284.1±4.0	249.5±4.6^a^	310.8±7.4^a^	220.0±7.7^a^
Blood glucose (mmol/l)	6.0±0.2	23.9±0.9^a^	6.4±0.2	23.0±1.2^a^

Injection refers to an intraperitoneal injection of alloxan monohydrate dissolved in normal saline to induce diabetes. Values are presented as the means ± SEM. FBS levels were measured before and after the experiments. The 'diabetic rats 7 days post-wounding' group indicates the group treated with arnebin-1.

a P<0.01 vs. non-diabetic rats.
